# Application of Improved Manta Ray Foraging Optimization Algorithm in Coverage Optimization of Wireless Sensor Networks

**DOI:** 10.1155/2022/3082933

**Published:** 2022-06-30

**Authors:** Fang Zhu, Wenhao Wang, Shan Li

**Affiliations:** School of Computer and Communication Engineering, Northeastern University at Qinhuangdao, Qinhuangdao 066004, China

## Abstract

For the shortcomings of the manta ray foraging optimization (MRFO) algorithm, like slow convergence speed and difficult to escape from the local optimum, an improved manta ray foraging algorithm based on Latin hypercube sampling and group learning is proposed. Firstly, the Latin hypercube sampling (LHS) method is introduced to initialize the population. It divides the search space evenly so that the initial population covers the whole search space to maintain the diversity of the initial population. Secondly, in the exploration stage of cyclone foraging, the Levy flight strategy is introduced to avoid premature convergence. Before the somersault foraging stage, the adaptive t-distribution mutation operator is introduced to update the population to increase the diversity of the population and avoid falling into the local optimum. Finally, for the updated population, it is divided into leader group and follower group according to fitness. The follower group learns from the leader group, and the leader group learns from each other through differential evolution to further improve the population quality and search accuracy. 15 standard test functions are selected for comparative tests in low and high dimensions. The test results show that the improved algorithm can effectively improve the convergence speed and optimization accuracy of the original algorithm. Moreover, the improved algorithm is applied to wireless sensor network (WSN) coverage optimization. The experimental results show that the improved algorithm increases the network coverage by about 3% compared with the original algorithm, and makes the optimized node distribution more reasonable.

## 1. Introduction

With the advancement and development of intelligent information technology, the scale and complexity of data are also increasing. Traditional numerical optimization methods are difficult to solve complex optimization problems, resulting in higher and higher calculation costs. In recent years, swarm-based intelligent optimization algorithms have been favored by many researchers because of their simplicity and high efficiency [1]. Swarm intelligence algorithms can effectively solve many complex optimization problems in the field of engineering, and are mainly used in network optimization [2], feature selection [3], image processing [4], automatic control [5], and other fields. In recent years, swarm intelligence optimization algorithms have been proposed, including butterfly optimization algorithm (BOA) [6], whale optimization algorithm (WOA) [7], sine cosine algorithm (SCA) [8], sparrow search algorithm (SSA) [9], marine predator algorithm (MPA) [10], African vultures optimization algorithm (AVOA) [11], manta ray foraging optimization (MRFO) algorithm [12], and so on.

The MRFO algorithm is a new swarm intelligence optimization algorithm proposed by Weiguo Zhao et al. in 2020. The inspiration of this algorithm is based on intelligent behaviors of manta rays. The foraging (optimization) process is divided into three stages, namely chain foraging, cyclone foraging, and somersault foraging. Compared with some classical intelligent algorithms and most of the above algorithms, it has higher convergence accuracy and faster optimization speed. Although MRFO has the above advantages, it still has the problems of easy premature convergence and falling into local optimum. In order to solve these problems, many researchers have improved the basic MRFO algorithm. Davut Izci et al. [13] introduced the opposition-based learning strategy into the population initialization, which improves the quality of the population to a certain extent, but convergence accuracy needs to be improved. Biqi Sheng et al. [14] proposed a balanced manta ray foraging optimization (BMRFO) algorithm. BMRFO introduces the Levy flight strategy in the cyclone foraging stage, and improves the flip factor. Although the algorithm's ability to jump out of the local optimum is improved, the convergence speed is not significantly improved. Oguz [15] introduces the chaotic map into the foraging behavior of MRFO, which improves the optimization performance of the algorithm, but the improvement ability was limited.

In order to better solve the problems and improve the optimization accuracy and convergence speed of the MRFO algorithm, this paper combines the Latin hypercube sampling (LHS) method with the group learning strategy, and introduces the Levy flight and adaptive t-distribution disturbance strategy. Therefore, an improved MRFO algorithm based on LHS and group learning (LGMRFO) is proposed. To verify the performance of the LGMRFO algorithm, 15 general test functions and 9 CEC2017 test suite functions are selected for low-dimensional and high-dimensional comparison tests.

Adaptive adjustment and deployment of sensor nodes in WSN can make them more evenly distributed in the detection area and have a higher coverage, so as to rationally allocate network space resources and better complete the tasks of environmental awareness and information acquisition. This is of great significance to improve network viability, improve network reliability, and save network construction costs. Generally, area coverage is the main criterion for evaluation. Optimized coordinate deployment of sensor nodes is carried out through optimization algorithm, and as few sensor nodes as possible are used to ensure the area coverage requirement and reduce the redundancy of sensor nodes. Therefore, in order to improve the poor coverage effect caused by unreasonable deployment of WSN nodes, the LGMRFO is applied to the coverage optimization problem of WSN. The experimental results further verify the effectiveness of the algorithm.

The rest of this paper is organized as follows. The MRFO algorithm is described in details in section “MRFO”. Section “Related Works” detailly introduces some intelligence optimization algorithms. Section “LGMRFO” describes the improved strategies for MRFO in this work. The performance of LGMRFO is evaluated by optimizing 24 test functions in section “Numerical Simulation Analysis”. Section “Coverage optimization of WSN Based on LGMRFO” presents the simulations and performance evaluation of LGMRFO for WSN coverage. At last, Section “Conclusion” summarizes this paper.

## 2. Related Works

Based on the source inspiration, the intelligence optimization algorithms can be divided into four classes of [16]: (a) physics-based, (b) math-based, (c) human-based, and (d) swarm-based. Physics-based methods tend to perceive the landscape as a physical phenomenon and move the search agents using formulae borrowed from physical rules or theories. The Archimedes optimization algorithm [17] is devised with inspirations from an interesting law of physics Archimedes' principle. An equilibrium optimizer (EO) [18] is inspired by control volume mass balance models used to estimate both dynamic and equilibrium states. Atomic orbital search (AOS) [19] is proposed based on some principles of quantum mechanics and the quantum-based atomic model. Transient search optimization (TSO) [20] is inspired by the transient behavior of switched electrical circuits that include storage elements.

Math-based algorithms are solely based on mathematical equations. They are not inspired by a specific natural phenomenon. Runge Kutta optimizer (RUN) [21] is designed according to the mathematical foundations of the Runge Kutta method. Gradient-based optimizer (GBO) [22] is inspired by the gradient-based Newton's method. The golden sine algorithm (Gold-SA) [23] is inspired by sine that is a trigonometric function. The arithmetic optimization algorithm (AOA) [24] utilizes the distribution behavior of the main arithmetic operators in mathematics. Weighted mean of vectors (INFO) [25] is an efficient optimization algorithm based on weighted mean of vectors.

Inspired by the social behaviors of human beings, a lot of optimization algorithms have been proposed. Political optimizer (PO) [26] is inspired by the multiphased process of politics. The group teaching optimization algorithm (GTOA) [27] simulated the impact of teachers on learners' output in the classroom. Queuing search (QS) [28] is inspired from human activities in queuing. Student psychology based optimization (SPBO) [29] is inspired by the psychology of the students who are trying to give more effort to improve their performance in the examination up to the level for becoming the best student in the class.

Swarm-based approaches imitate the social behavior and communications within a group of species of animals, plants, or other living things. These approaches have gained increasing popularity in terms of both application and new algorithm development. Some of the recently proposed algorithms that can be categorized under this approach are slime mould algorithm (SMA) [30], hunger games search (HGS) [31], Harris hawks optimization (HHO) [32], moth search algorithm (MSA) [33], monarch butterfly optimization (MBO) [34], golden eagle optimizer (GEO) [35], and tuna swarm optimization (TSO) [36].

Compared with these three types, swarm-based algorithms have superiority over other three types of algorithms. Manta ray foraging optimization (MRFO), with few adjustable parameters, is easy to implement, which in turn makes it very potential for applications in many engineering fields. So, this paper improves the manta ray foraging optimization (MRFO) algorithm named MRFO based on Latin hypercube sampling and group learning (LGMRFO). MRFO falls into the fourth class of optimization algorithms, as it originates from swarm behavior of manta rays (a kind of sea animal).

## 3. MRFO

MRFO updates the individual position by three foraging behaviors, including chain foraging, cyclone foraging, and somersault foraging. The mathematical models are described below.

### 3.1. Chain Foraging

Manta rays' line up head-to-tail and form a foraging chain. In each iteration, each individual is updated by the best solution found so far and the solution in front of it. This mathematical model of chain foraging is represented as follows:

(1) $$\begin{array}{c} x_{i}^{d}\left(t+1\right)=\left\{\begin{array}{cc} x_{i}^{d}\left(t\right)+r\cdot \left(x_{\text{best}}^{d}\left(t\right)-x_{i}^{d}\left(t\right)\right)+\alpha \cdot \left(x_{\text{best}}^{d}\left(t\right)-x_{i}^{d}\left(t\right)\right), & i=1,\\ x_{i}^{d}\left(t\right)+r\cdot \left(x_{i-1}^{d}\left(t\right)-x_{i}^{d}\left(t\right)\right)+\alpha \cdot \left(x_{\text{best}}^{d}\left(t\right)-x_{i}^{d}\left(t\right)\right), & i=2,\ldots ,N, \end{array}\right. \end{array}$$

(2) $$\begin{array}{c} \alpha =2\cdot r\cdot \sqrt{\left|\log\left(r\right)\right|}, \end{array}$$

where, *x*_*i*_^*d*^(*t*) is the position of ith individual at t-th iteration, *r* is a random vector within the range of [0, 1], *α* is a weight coefficient, *x*_best_^*d*^(*t*) is the plankton with high concentration (the best solution found so far), and N denotes the population size.

### 3.2. Cyclone Foraging

When manta rays find plankton in deep water, they form a long foraging chain and swim towards the food by a spiral. In the cyclone foraging behavior of manta rays, in addition to spirally move towards the food, each manta ray swims towards the one in front of it. The mathematical model of the exploitation stage of cyclone foraging behavior can be calculated by the following formula:

(3) $$\begin{array}{c} x_{i}^{d}\left(t+1\right)=\left\{\begin{array}{cc} x_{\text{best}}^{d}+r\cdot \left(x_{\text{best}}^{d}\left(t\right)-x_{i}^{d}\left(t\right)\right)+\beta \cdot \left(x_{\text{best}}^{d}\left(t\right)-x_{i}^{d}\left(t\right)\right), & i=1,\\ x_{\text{best}}^{d}+r\cdot \left(x_{i-1}^{d}\left(t\right)-x_{i}^{d}\left(t\right)\right)+\beta \cdot \left(x_{\text{best}}^{d}\left(t\right)-x_{i}^{d}\left(t\right)\right), & i=2,\ldots ,N, \end{array}\right. \end{array}$$

(4) $$\begin{array}{c} \beta =2e^{r_{1}\left(T-t+1/T\right)}\cdot \sin\left(2\pi r_{1}\right), \end{array}$$

where *β* is a weight factor, *T* is the maximum number of iterations, and *r*_1_ is a rand number in [0, 1].

In equation (3), MRFO focuses on local exploitation. In addition, by taking the random position in the search space as the reference position, this behavior can also be used to improve the exploration mechanism of the algorithm. The mathematical model is as follows:

(5) $$\begin{array}{c} x_{\text{rand}}^{d}=Lb^{d}+r\cdot \left(Ub^{d}-Lb^{d}\right),\\ x_{i}^{d}\left(t+1\right)=\left\{\begin{array}{cc} x_{\text{rand}}^{d}+r\cdot \left(x_{\text{rand}}^{d}-x_{i}^{d}\left(t\right)\right)+\beta \cdot \left(x_{\text{rand}}^{d}-x_{i}^{d}\left(t\right)\right), & i=1,\\ x_{\text{rand}}^{d}+r\cdot \left(x_{i-1}^{d}\left(t\right)-x_{i}^{d}\left(t\right)\right)+\beta \cdot \left(x_{\text{rand}}^{d}-x_{i}^{d}\left(t\right)\right), & i=2,\ldots ,N, \end{array}\right. \end{array}$$

where *x*_rand_^*d*^ is a random position produced in the search space, *Lb*^*d*^ and *Ub*^*d*^ are the lower and upper limits of the dth dimension, respectively.

### 3.3. Somersault Foraging

In this foraging behavior, the position of food is regarded as a pivot. Each individual tends to swim to and from around the pivot and somersault to a new position. The mathematical model can be created as follows:

(6) $$\begin{array}{c} x_{i}^{d}\left(t+1\right)=x_{i}^{d}\left(t\right)+S\cdot \left(r_{2}\cdot x_{\text{best}}^{d}-r_{3}\cdot x_{i}^{d}\left(t\right)\right),\;i=1,\ldots ,N, \end{array}$$

where S is the somersault factor that decides the somersault range of manta rays and *S*=2, *r*_2_ and *r*_3_ are two random number in [0, 1].

MRFO balances the ability of global exploration and local exploitation by controlling the change in *t*/*T*, where, *t* is the current number of iterations and *T* is the maximum number of iterations. When *t*/*T* < rand, selecting the current optimal position as the reference position for global exploration behavior. When *t*/*T* ≥ rand, taking the optimal individual as the reference point, it focuses on the local exploitation ability of the algorithm.

## 4. LGMRFO

In order to improve the performance of MRFO, this paper improves it in three aspects: Firstly, the LHS method is used to initialize the population to enhance the diversity of the population; Secondly, in the exploration stage of cyclone foraging, Levy flight strategy is introduced to accelerate the convergence speed. Before the somersault foraging, an adaptive t-distribution mutation operator is added to update the population position to avoid falling into local optimization; Finally, the group learning strategy is set to improve the optimization accuracy of the algorithm.

### 4.1. LHS Method Population Initialization Strategy

In the basic MRFO, the initial population is generated in a random way. The initial population generated by this method is often unevenly distributed or even overlaps individuals, which reduces the optimization performance of the algorithm to a certain extent. The LHS method is a multidimensional stratified sampling technology proposed by McKay et al. [37], which has the following advantages compared with simple random sampling method.

1. The sampling points generated by LHS can achieve full space coverage and can be evenly distributed in the search space;
2. LHS has better robustness and stability.

Therefore, in order to enhance the diversity of the initial population and improve the performance, we adopt the LHS method to initialize the population.

Assuming that N initial individuals are generated in the d-dimensional space, the specific steps to initialize the population with the LHS method are as follows:

 
*Step 1.* Firstly, the population size N and dimension d are determined.
 
*Step 2.* Determine the interval for individual x as [lb, ub], where lb and ub are the lower and upper bounds of the variable x, respectively.
 
*Step 3.* Divide the interval of variable x into N equal small intervals.
 
*Step 4.* Randomly select a point in each subinterval of each dimension.
 
*Step 5.* Combine the extracted points of each dimension to form initial population.

Figure 1 and 2 are sample point maps generated by the LHS method and simple random sampling method, respectively, where the sampling size is 20 and dimension is 2. It can be seen that the sample points generated by the LHS method can be more evenly distributed in the search space. Therefore, using the LHS method to initialize the population of the MRFO algorithm, it can make the population position evenly distributed in the search space, and enhance the population diversity to improve the convergence performance of the algorithm.

### 4.2. Mutation Strategy

#### 4.2.1. Levy Flight

In some cases, due to the random individual selection in each iteration, premature convergence may occur, thereby increasing the running time, so different mechanisms can be used to improve the MRFO algorithm. This paper uses the Levy flight mechanism [38] for local disturbance, the mechanism is based on random walk behavior, and the mathematical model is as follows:

(7) $$\begin{array}{c} \text{Levy}\left(\lambda \right)=\frac{u}{{\left|v\right|}^{-\lambda }}, \end{array}$$

where *u* and *v* come from the normal distribution, i.e.,

(8) $$\begin{array}{c} u∼N\left(0,\sigma_{u}^{2}\right)\;v∼N\left(0,\sigma_{v}^{2}\right). \end{array}$$

The values of *σ*_*u*_ and *σ*_*v*_ are as follows:

(9) $$\begin{array}{c} \sigma_{u}={\left\{\frac{\Gamma \left(1+\lambda \right)\sin\left(\pi \lambda /2\right)}{\Gamma \left(1+\lambda /2\right)\lambda 2^{\lambda -1/2}}\right\}}^{1/\lambda },\;\sigma_{v}=1, \end{array}$$

where Γ is the standard gamma function.

The position update formula of the cyclone foraging exploration stage with the addition of Levy flight strategy is as follows:

(10) $$\begin{array}{c} x_{i}^{d}\left(t+1\right)=\left\{\begin{array}{cc} x_{\text{rand}}^{d}+\text{Levy}\left(\lambda \right)⊗\left[r\cdot \left(x_{\text{rand}}^{d}-x_{i}^{d}\left(t\right)\right)+\beta \cdot \left(x_{\text{rand}}^{d}-x_{i}^{d}\left(t\right)\right)\right], & i=1,\\ x_{\text{rand}}^{d}+\text{Levy}\left(\lambda \right)⊗\left[r\cdot \left(x_{i-1}^{d}\left(t\right)-x_{i}^{d}\left(t\right)\right)+\beta \cdot \left(x_{\text{rand}}^{d}-x_{i}^{d}\left(t\right)\right)\right], & i=2,\ldots ,N, \end{array}\right. \end{array}$$

where ⊗ denotes point-to-point multiplication.

#### 4.2.2. Adaptive t-Distribution

T-distribution is also called student distribution [39], and its distribution state is closely related to degrees of freedom. In order to enhance the diversity of the population and avoid falling into local optimum, this paper introduces the adaptive t-distribution strategy to disturb manta ray population before the somersault foraging behavior. The calculation formula is as follows:

(11) $$\begin{array}{c} x_{\text{new}}=x_{\text{old}}+x_{\text{old}}\cdot t\left(\text{iter}\right), \end{array}$$

where *x*_old_ is the original individual, *x*_new_ is the new individual after mutation, and *t*(iter) is the t-distribution with the current iteration number iter as the degree of freedom.

In the early stage of the iteration, the degree of freedom is small (the number of iterations is small), and t-distribution is similar to Cauchy distribution. At this time, the update step size is larger, which can expand the search field of the individual and improve the global exploration ability. In the middle and later iteration, the degree of freedom gradually increases, and the performance of t-distribution is similar to Gauss distribution. At this time, the update step size is smaller, which helps the algorithm to search around the current individual neighbourhood, and the algorithm has better local exploitation ability.

### 4.3. Group Learning Strategy

In the process of algorithm evolution, some individuals may reach the optimal position, and the fitness value of others may become more worse. In order to overcome this defect, inspired by the salp swarm algorithm (SSA) [40], individuals with poor location need to learn foraging skills from individuals with good location. Based on this idea, a group learning strategy is proposed. The population after somersault foraging is evenly divided into two groups according to the fitness value. The group with better fitness is called the leader group, and the group with poor fitness is called the follower group.

#### 4.3.1. Leader Group Learning Strategy

The differential evolution (DE) algorithm [41] has a good effect in solving complex optimization problems. In this paper, the differential evolution strategy is used to generate a new leader group individual, and the greedy strategy is used to select the optimal individual. The specific mathematical model is as follows:

(12) $$\begin{array}{c} x_{\text{new}}=x_{\text{best}}^{\prime }+F\cdot \left(x_{m}-x_{n}\right), \end{array}$$

where *x*_new_ is a new individual produced by mutation; *x*_best_′ is the optimal individual *x*_best_ new individuals generated by randomly sorting dimensions; *F* is the scaling factor, and *F*=0.5; *x*_*m*_ and *x*_*n*_ are two different leaders randomly selected from the leadership group, which are different from the current individual. The new individual generated by this strategy needs to be compared with the original individual, and the individual with better fitness should be selected as the current individual.

Compared with the mutation of whole individuals, this strategy has stronger selectivity, which can effectively enhance the local mining performance and improve the convergence accuracy of the algorithm.

#### 4.3.2. Follower Group Learning Strategy

Each follower in the follower group learns from the average of the two leaders. The mathematical model is described as follows:

(13) $$\begin{array}{c} x_{\text{follower}}^{i\_\text{new}}=\frac{\left(x_{\text{leader}}^{i}+x_{\text{leader}}^{i+1}\right)}{2}, \end{array}$$

where *x*_follower_^*i*_new^ refers to the new individual generated after the *i*th individual of the following group learns from the leading group, *x*_leader_^*i*^ represents the *i*th individual of the leadership group. The new follower individual needs to be compared with the original follower individual, and the individual with a better fitness value is selected as the current follower individual.

By learning from the leader group, the follower group can greatly improve the fitness, realize the conversion from follower to leader, and then improve the convergence speed of the algorithm.

### 4.4. LGMRFO Algorithm Implementation Steps

The specific implementation steps of LGMRFO algorithm are as follows:

 
*Step 1.* Set the relevant parameters: population size N, variable dimension *D*, maximum number of iterations *T*, and initialize the population position by the LHS method.
 
*Step 2.* The fitness value of each individual is calculated, and the initial optimal individual position and its optimal fitness value are obtained according to the fitness value.
 
*Step 3.* Enter the algorithm iteration process. When rand ≥ 0.5, chain foraging is performed and updates the individual position according to equation (1); Otherwise, cyclone foraging is performed, when *t*/*T* < rand, the individual enters the exploration stage, introduces Levy flight strategy, and updates the individual position according to equation (10), when *t*/*T* < rand, the individual enters the development stage and updates the individual position according to equation (3).
 
*Step 4.* Before performing somersault foraging behavior, an adaptive t-distribution strategy is added, the individual position is updated according to equation (11), and the current individual is greedily selected.
 
*Step 5.* Perform somersault foraging behavior according to equation (6).
 
*Step 6.* The group learning strategy is implemented, that is, the updated population is divided into a leading group and a following group according to the fitness value, and new individuals are generated by learning from equations (12) and (13), respectively. If the fitness becomes better after learning, the current individual position will be updated, otherwise, it will not be updated.
 
*Step 7.* Update the optimal location and its optimal fitness value of each generation.
 
*Step 8.* Judge whether the algorithm meets the iteration conditions. If so, the algorithm terminates; Otherwise, go to Step 3.

The pseudocode of LGMRFO is shown in Algorithm 1.

### 4.5. Time Complexity of the LGMRFO

The overall time complexity of MRFO is given as

(14) $$\begin{array}{c} O\left(\text{MRFO}\right)=O\left(T\left(O\left(\text{cyclone foraging}+\text{chain foraging}\right)\right)\right)+O\left(\text{somersault foraging}\right),\\ O\left(\text{MRFO}\right)=O\left(T\left(nd+nd\right)\right)=O\left(Tnd\right), \end{array}$$

where, *T* is the maximum number of iterations, *n* is the number of individuals, and *d* is the number of variables.

LGMRFO proposed that in this paper only increases the computational complexity in adaptive t-distribution and group learning. Therefore, the overall time complexity of LGMRFO is given as

(15) $$\begin{array}{c} O\left(\text{LGMRFO}\right)=O\left(\text{MRFO}\right)+O\left(T\left(\text{O}\left(\text{adaptive }t-\text{distribution}\right)+O\left(\text{group learning}\right)\right)\right),\\ O\left(\text{LGMRFO}\right)=O\left(\text{MRFO}\right)+O\left(T\left(nd+nd\right)\right)=O\left(Tnd\right). \end{array}$$

This shows that the time complexity of LGMRFO is consistent with that of MRFO.

## 5. Numerical Simulation Analysis

24 test functions are chosen and experimentally tested with five algorithms for finding the minimal value of the function: BOA, WOA, SCA, SSA (sparrow search algorithm), and MRFO, in order to evaluate the effectiveness of the proposed LGMRFO algorithm. Refer to the corresponding original literature for specific parameter settings.

### 5.1. Test Functions

1. General functions: Single*-*peaked functions have only one global best point and no local extreme points, while the test functions F1 to F4 are multidimensional single*-*peaked functions, F5 to F12 are high-dimensional multipeaked functions, and F13 to F15 are three fixed-dimensional multipeaked functions. The multipeak function has numerous local extremum points, which are utilized to observe the performance of the function jumping out of local extremum points in different dimensions from two high-dimensional views.  Table 1 shows the precise function details.
2. CEC2017 test suite functions: In order to further test the performance of LGMRFO, this paper selects some CEC2017 test suite functions [42] for testing, which are CF2, CF4, CF7, CF8, CF10, CF15, CF17, CF20, and CF24, respectively, with *D* = 30 and Range ∈ [−100, 100].

### 5.2. Results Evaluation of General Functions

Simulation and comparison experiments of six algorithms were conducted in the Matlab R2018a environment. To avoid excessive chance errors, each benchmark function was chosen to run 30 times independently in the experiments, and the optimal value, the worst value, the average value, and standard deviation were used as evaluation indexes, and the population size was set to 30 and the maximum number of iterations was 500. Black highlights the greatest outcomes. F13 to F15 (fixed-dimensional multipeak function), *D* = 50 (low-dimensional), and *D* = 500 (high-dimensional) functions F1 to F12, respectively, are used to test and assess the algorithm.

The iterative convergence curves of six algorithms at 500 dimensions under four single peak test functions, eight multipeak function test functions, and three fixed-dimension test functions are plotted in this research due to the article length constraint, as shown in Figure 3.

#### 5.2.1. Multipeak Function Test with Fixed Dimensions

Table 2 shows the test results for the three fixed-dimension multipeak functions from F13 to F15. Table 2 and Figures 3(e) and 3(f) show that LGMRFO has faster convergence and better optimization-seeking accuracy than other algorithms, and its standard deviation is the smallest, indicating that it is more stable. The standard deviation reflects the algorithm's stability in solving, so LGMRFO is more stable.

#### 5.2.2. Evaluation of Low-Dimensional Functions

Table 3 shows a comparison of the algorithm's function test results in 50 dimensions. Both LGMRFO and basic MRFO can meet the theoretical optimal value in the single-peak low-dimensional function test, as shown in Table 3, and standard deviation is 0. This indicates that LGMRFO's optimization-seeking ability is more stable than other algorithms, and LGMRFO's convergence speed is significantly faster than other intelligent algorithms, including MRFO, indicating that the improvement strategy has significantly improved MRFO's convergence performance. Table 2 shows that LGMRFO can also get greater accuracy solutions in the multipeak low-dimensional function test, especially for functions F5, F6, F7, F8, and F10. Although the average solutions of functions F9, F11, and F12 do not approach the theoretical ideal value, LGMRFO's overall convergence performance ranks 2nd, 1st, and 2nd, respectively, when compared to other algorithms. The other algorithms have a better chance of escaping the local optimum. Except for functions F9 and F12, LGMRFO has the smallest standard deviation among the other functions, hence its robustness is higher in terms of stability.

#### 5.2.3. Evaluation of High-Dimensional Functions

Table 3 shows a comparison of the algorithms' outcomes in the 500-dimensional function test. It is obvious from a comparison of the experimental findings of the low-dimensional function test that LGMRFO gets better outcomes in terms of both search accuracy and convergence speed. The increase in dimensionality of the function from a low-dimensional to a high-dimensional function will affect the algorithm's convergence performance. Table 3 shows that both LGMRFO and basic MRFO approach the theoretical optimum with a standard deviation of 0 in the single peaked high-dimensional test function. This indicates that LGMRFO and MRFO are stable, and the convergence speed of LGMRFO is faster than other algorithms, as shown in Figures 3(a)∼3(d), demonstrating the superiority of the improved strategy, whereas the convergence results of other compared algorithms are worse than the low-dimensional function. The standard deviation is also higher than in the low dimension, indicating that the other comparison algorithms are less robust on single-peaked high-dimensional functions; LGMRFO ranks first in the multipeaked high-dimensional function test, except for function F9; and LGMRFO ranks first in the low-dimensional multipeaked function F12, indicating that the improvement strategy in higher ability. In terms of convergence performance under high-dimensional functions, LGMRFO still outperforms the other five techniques.

### 5.3. Results Evaluation of CEC2017 Test Suite Functions

Table 4 shows a comparison of the algorithms' outcomes in some CEC2017 test suite functions.  Figure 4 shows the average convergence curves of some CEC2017 test suite functions. Therefore, LGMRFO achieves the best results in CF2, CF4, CF7, CF8, CF10, CF17, and CF20. It shows that the overall performance of LGMRFO is powerful so that it can perform a smoother transition between exploration and exploration trends.

### 5.4. Wilcoxon Rank Sum Test

The Wilcoxon rank sum test [43] is a nonparametric statistical test that is performed to see if the LGMRFO method is significantly different from others. As a result, the results of the five algorithms were tested 30 times independently on 15 test functions and 9 CEC2017 functions as samples, and the Wilcoxon rank sum test was used to determine the significant difference between the solution results of the five compared algorithms and the LGMRFO solution results for the 50 and 500-dimensional, fixed-dimensional functions, and 9 CEC2017 functions, respectively. Tables 5–7 show the outcomes of the tests.

The null hypothesis is rejected when *P* < 0.05 indicates that the two algorithms are statistically different, whereas *P* > 0.05 implies that the two algorithms provide equivalent search results, according to the literature [44]. “NaN” implies that the associated algorithm searches for theoretical optimal solution, hence this hypothesis test is not applicable. In the 50-dimensional instance, the LGMRFO algorithm performs much better than the other examined algorithms, with the exception of MRFO, whereas in the 500-dimensional situation, the LGMRFO method performs significantly better than the 50-dimensional one. In the 9 CEC2017 functions situation, among the 45 data sets, 42 are less than 0.05, comprising 93.3% of the total data. This shows that LGMRFO has statistical advantages over the other competitive algorithms. In conclusion, LGMRFO outperforms MRFO, SSA, SCA, WOA, and BOA by a statistically significant margin, indicating that the LGMRFO algorithm is statistically superior.

## 6. Coverage Optimization of WSN Based on LGMRFO

### 6.1. WSN Node Coverage Model

The Boolean measurement model and the probabilistic measurement model are the two basic types of WSN node coverage models [45]. In this research, we calculate network coverage using the more standard Boolean model.

Assume that in a square WSN monitoring region with a side length of *L*, N isomorphic sensor nodes are randomly distributed. Assume that the set of nodes is V={*v*_1_, *v*_2_,…, *v*_*N*_}, with node *v*_*i*_'s location coordinates being (*x*_*i*_, *y*_*i*_), and each node's sensing radius being *R*_*s*_. The area is discretized into *m* × *n* target grid points to be covered to make the calculation easier, and the set of target points is indicated as *u*_*j*_=(*x*_*j*_, *y*_*j*_), *j* ∈ {1,2,…, *m* × *n*}. The distance between the sensor node and the target point is specified as

(16) $$\begin{array}{c} d\left(v_{i},u_{j}\right)=\sqrt{{\left(x_{i}-x_{j}\right)}^{2}+{\left(y_{i}-y_{j}\right)}^{2}}. \end{array}$$

The target point has been covered if there is a node whose distance from the target point is less than or equal to the sensing radius *R*_*s*_. According to the Boolean model, the chance that the sensor node *v*_*i*_ detects the target location is defined as

(17) $$\begin{array}{c} p\left(v_{i},u_{j}\right)=\left\{\begin{array}{cc} 0, & d\left(v_{i},u_{j}\right)>R_{s},\\ 1, & d\left(v_{i},u_{j}\right)\leq R_{s}. \end{array}\right. \end{array}$$

When the target point is sensed by more than one sensor, the joint sensing probability of the target point is defined as

(18) $$\begin{array}{c} p\left(V,u_{j}\right)=1-\prod_{i=1}^{N}\left[1-p\left(v_{i},u_{j}\right)\right]. \end{array}$$

The area network coverage is calculated by multiplying the sum of the total perceived probability of target points covered by a set of nodes by the entire number of target points in the area.

(19) $$\begin{array}{c} R_{\mathrm{cov}}=\frac{\sum_{j=1}^{m\times n}p\left(V,u_{j}\right)}{m\times n}. \end{array}$$

As a result, the WSN coverage optimization issue can be defined as the coverage of complete target grid points by N sensor nodes on the monitoring area using an optimization technique, which can then be turned into a single objective optimization problem that maximizes equation. (17), i.e.,

(20) $$\begin{array}{c} \max\left(\frac{\sum_{j=1}^{m\times n}p\left(V,u_{j}\right)}{m\times n}\right). \end{array}$$

### 6.2. Analysis of Simulation

Two sets of experiments are used in this work to verify the efficiency of LGMRFO on WSN coverage optimization. As stated in Table 8, the experimental settings have been set.

Figure 5 shows the results of sensor area coverage after algorithm optimization. The distribution at 30 nodes is shown in Figure 5(a) and 5(b), with MRFO covering 82.43 percent of the nodes and LGMRFO covering 84.78 percent. In the monitoring region, there are still coverage blind spots, and node overlapping coverage is more evident, as shown in Figure 5(a), but the optimized nodes in Figure 5(b) are more uniformly distributed. Figures 5(c) and 5(d) show the coverage results when 35 nodes are installed. After MRFO optimization, the coverage rate is 89.43%, yet there are coverage blind patches near the monitoring area's edge. After LGMRFO optimization, the coverage rate is 92.62%, and the node overlapping area is greatly reduced.

Table 9 shows the coverage of MRFO and LGMRFO running independently for 20 times and each operation iteration for 500 times, respectively. As can be seen from Table 9, LGMRFO's final and initial coverage are higher than those of the MRFO algorithm, indicating that the LHS method's enhanced strategy and location update improve the algorithm's search accuracy.

The average coverage iteration curves are given in Figure 6. LGMRFO coverage in the middle of iteration is slightly lower than MRFO at 30 nodes in Figure 6(a), which is owing to the premature maturity produced by MRFO converging too quickly. LGMRFO gradually surpasses MRFO after 300 iterations, suggesting that MRFO has entered the local optimum, whereas LGMRFO jumps out of the local optimum and optimization accuracy improves, demonstrating that the group learning technique is effective. The population's health (node distribution) has improved, and the coverage rate has continuously increased. LGMRFO's coverage is greater than MRFO's when 35 nodes are deployed, which corresponds to an increase in individual dimension, and both the convergence speed and coverage are much greater than the MRFO algorithm's average optimization result.

In summary, by comparing the experimental results of deploying different numbers of nodes, LGMRFO achieves higher average network coverage under the same conditions, and the node layout is more reasonable, resulting in fewer coverage blind areas and overlapping areas, proving the effectiveness of the improved strategy.

## 7. Conclusion

To overcome the inadequacies of the manta ray foraging optimization method in terms of optimization accuracy, this work offers an improved manta ray foraging optimization algorithm (LGMRFO). Firstly, to improve the quality of the initial population, the LHS method is used to homogenize the population position distribution. Secondly, the Levy flight and adaptive t-distribution variation strategies are used before the cyclone foraging exploration phase and somersault foraging behavior, respectively, so as to improve the algorithm's ability to jump out of the local optimum. Finally, a group learning strategy is used for the updated population. On 24 typical test functions, the LGMRFO algorithm is compared to the other five algorithms, and the method significance level is validated using the Wilcoxon rank sum test. LGMRFO greatly enhances convergence speed, optimization-seeking accuracy, and global optimization capability, according to the findings of the experiments. Finally, on the WSN coverage optimization problem, LGMRFO is compared to MRFO, and the experimental findings support the usefulness of the proposed improvement strategies.

As future challenges, different applications other than WSN coverage optimization of LGMRFO can be explored and its capabilities in dealing with difficult test problems can be examined. Besides, new configurations of this algorithm can be considered as other researchers may have different viewpoints on the presented methodology.

## Figures and Tables

**Figure 1:** Samples distribution map based on the LHS method.

**Figure 2:** Samples distribution map based on the random method.

**Figure 3:** Average convergence curves of 500 dimensional partial functions and fixed-dimensional functions F14 and F15. (a) F1 (b) F2. (c) F5 (d) F6. (e) F14 (f) F15.

**Figure 4:** Average convergence curves of some CEC2017 test suite functions. (a) CF2. (b) CF4. (c) CF7 (d) CF8. (e) CF10. (f) CF15. (g) CF17. (h) CF20. (i) CF24.

**Figure 5:** Node distribution before and after algorithm optimization: (a) Coverage result of MRFO (*N* = 30), (b) Coverage result of LGMRFO (*N* = 30), (c) Coverage result of MRFO (*N* = 35), and (d) Coverage result of LGMRFO (*N* = 35).

**Figure 6:** Average coverage iteration curve: (a) Average coverage iteration curve (*N* = 30) and (b) Average coverage iteration curve (*N* = 35).

**Algorithm 1:** LGMRFO Algorithm.

**Table 1:** Test function information.

No.	Function name	Function formula	D	Range	Optimum
F1	Bent cigar	F1(*x*) = *x*_1_^2^+10^6^∑_*i*=2_^*D*^*x*_*i*_^2^	50/500	[−100, 100]	0
F2	Sum of different power	F2(*x*) = ∑_*i*=1_^*D*^|*x*_*i*_|^*i*+1^	50/500	[−100, 100]	0
F3	Zakharov	F3(*x*) = ∑_*i*=1_^*D*^*x*_*i*_^2^+(∑_*i*=1_^*D*^0.5*x*_*i*_)^2^+(∑_*i*=1_^*D*^0.5*x*_*i*_)^4^	50/500	[−100, 100]	0
F4	High conditioned	F4(*x*) = ∑_*i*=1_^*D*^(10^6^)^*i* − 1/*D*−1^*x*_*i*_^2^	50/500	[−100, 100]	0
F5	Griewank's	F5(*x*) = $\sum_{i=1}^{d}x_{i}^{2}/4000-\overset{D}{\underset{i=1}{\prod }}\cos\left(x_{i}/\sqrt{i}\right)+1$	50/500	[−100, 100]	0
F6	Rastrigin	F6(*x*) = ∑_*i*=1_^*D*^(*x*_*i*_^2^ − 10cos(2*πx*_*i*_)+10)	50/500	[−100, 100]	0
F7	Expanded Schaffer's	F7(*x*) = ∑_*i*=1_^*D*−1^*y*(*x*_*i*_, *x*_*i*+1_)+*y*(*x*_*D*_, *x*_1_)			
		*y*(*u*, *v*) = $0.5+\left(\sin^{2}\left(\sqrt{u^{2}+v^{2}}\right)-0.5\right)/{\left(1+0.001\left(u^{2}+v^{2}\right)\right)}^{2}$	50/500	[−100, 100]	0
F8	Noncontinuous rotated Rastrigin's	F8(*x*) = ∑_*i*=1_^*D*^[*y*_*i*_^2^ − 10cos(2*πy*_*i*_)+10]*y*_*i*_ = $\left\{\begin{array}{c} x_{i}\;\left|x_{i}\right|<0.5\\ \text{round}\left(2x_{i}\right)/2\;\left|x_{i}\right|\geq 0.5 \end{array}\right.$	50/500	[−100, 100]	0
F9	Rosenbrock's	F9(*x*) = ∑_*i*=1_^*D*−1^[100(*x*_*i*_^2^ − *x*_*i*+1_)^2^+(*x*_*i*_ − 1)^2^]	50/500	[−100, 100]	0
F10	*Discus*	F10(*x*) = 10^6^*x*_1_^2^+∑_*i*=1_^*D*^*x*_*i*_^2^	50/500	[−100, 100]	0
F11	Ackley	F11(*x*) = −20exp(−0.21/*D*∑_*i*=1_^*D*^*x*_*i*_^2^) − exp(1/*D*∑_*i*=1_^*D*^cos(2*πx*_*i*_))+20+*e*	50/500	[−100, 100]	0
F12	Schaffer's F7	F12(*x*) = ${\left[1/D-1\sum_{i=1}^{D-1}\left(\sqrt{s_{i}}\times \left(\sin\left(50s_{i}^{0.2}\right)+1\right)\right)\right]}^{2}$$s_{i}=\sqrt{x_{i}^{2}+x_{i+1}^{2}}$	50/500	[−100, 100]	0
F13	Foxholes	F13(*x*) = (1/500+∑_*j*=1_^25^1/*j*+∑_*i*=1_^2^(*x*_*i*_ − *a*_*ij*_)^6^)^−1^	2	[−65, 65]	1
F14	Schkel	F14(*x*) = −∑_*i*=1_^10^[(*X* − *a*_*i*_)(*X* − *a*_*i*_)^*T*^+*c*_*i*_]^−1^	4	[0, 10]	−10.5363
F15	Six-hump camel	F15(*x*) = 4*x*_1_^2^ − 2.1*x*_1_^4^+1/3*x*_1_^6^+*x*_1_*x*_2_ − 4*x*_2_^2^+4*x*_2_^4^	2	[−5, 5]	−1.0316

**Table 2:** Comparison of test results for fixed-dimensional function F13–F15.

Function	Algorithm	Best	Worst	Average	Std. Deviation
F13	BOA	0.9980	3.0050	1.2986	0.6261
	WOA	0.9980	10.7632	3.0888	3.5685
	SCA	0.9980	2.9821	1.7922	0.9882
	SSA	0.9980	12.6705	7.3556	5.7991
	MRFO	0.9980	0.9980	0.9980	1.01*E − *16
	LGMRFO	0.9980	0.9980	0.9980	9.22*E − *17

F14	BOA	−5.4578	−4.0632	−4.5494	0.2656
	WOA	−10.1531	−2.6283	−7.6042	2.8176
	SCA	−7.8812	−0.4973	−3.2410	2.0496
	SSA	−10.1532	−5.0552	−9.2006	1.9674
	MRFO	−10.1532	−5.0552	−8.7937	2.2930
	LGMRFO	−10.1532	−10.1532	−10.1532	6.33*E − *15

F15	BOA	−1.0316	−1.0287	−1.0307	8.58*E − *04
	WOA	−1.0316	−1.0316	−1.0316	2.01*E − *09
	SCA	−1.0316	−1.0316	−1.0316	3.96*E − *05
	SSA	−1.0316	−1.0316	−1.0316	6.39*E − *16
	MRFO	−1.0316	−1.0316	−1.0316	6.52*E − *16
	LGMRFO	−1.0316	−1.0316	−1.0316	5.61*E − *16

**Table 3:** Comparison of test results under different dimensions for function F1–F12.

Function	Algorithm	*D* = 50				*D* = 500			
		Best	Worst	Average	Std	Best	Worst	Average	Std

F1	BOA	1.38*E − *11	1.68*E − *11	1.55*E − *11	8.44*E − *13	1.45*E − *11	1.76*E − *11	1.60*E − *11	9.61*E − *13
	WOA	1.08*E − *79	1.32*E − *63	7.38*E − *65	2.86*E − *64	9.70*E − *81	2.86*E − *61	1.11*E − *62	5.23*E − *62
	SCA	1.01 E+07	3.24 E+09	8.14 E+08	8.47*E + *08	6.92*E + *10	3.38*E + *11	2.03*E + *11	7.12*E + *10
	SSA	0	1.20*E − *60	4.01*E − *62	2.19*E − *61	1.74*E − *248	2.91*E − *54	9.69*E − *56	5.31*E − *55
	MRFO	0	0	0	0	0	0	0	0
	LGMRFO	0	0	0	0	0	0	0	0

F2	BOA	6.27*E + *74	9.03*E + *89	8.05*E + *88	2.18*E + *89	Inf	Inf	Inf	NaN
	WOA	4.34*E − *112	2.54*E − *82	9.08*E − *84	4.65*E − *83	Inf	Inf	Inf	NaN
	SCA	2.41*E + *24	4.86*E + *48	1.65*E + *47	8.87*E + *47	Inf	Inf	Inf	NaN
	SSA	0	2.99*E − *37	9.96*E − *39	5.46*E − *38	0	7.82*E − *44	2.61*E − *45	1.43*E − *44
	MRFO	0	0	0	0	0	0	0	0
	LGMRFO	0	0	0	0	0	0	0	0

F3	BOA	1.11*E − *11	1.46*E − *11	1.28*E − *11	8.41*E − *13	1.10*E − *11	1.49*E − *11	1.34*E − *11	8.32*E − *13
	WOA	6.01*E + *04	1.47*E + *05	9.47*E + *04	1.83*E + *04	1.54*E + *06	1.86*E + *06	1.64*E + *06	6.22*E + *04
	SCA	2.643*E + *03	2.81*E + *04	1.28*E + *04	6.33*E + *03	2.98*E + *05	8.34*E + *05	5.59*E + *05	1.31*E + *05
	SSA	5.52*E − *169	1.24*E − *74	6.94*E − *76	2.68*E − *75	0	1.48*E − *61	4.95*E − *63	2.71*E − *62
	MRFO	0	0	0	0	0	0	0	0
	LGMRFO	0	0	0	0	0	0	0	0

F4	BOA	1.20*E − *11	1.68*E − *11	1.50*E − *11	9.51*E − *13	1.43*E − *11	1.75*E − *11	1.59*E − *11	8.93*E − *13
	WOA	4.59*E − *79	2.42*E − *66	8.32*E − *68	4.41*E − *67	2.65*E − *77	6.99*E − *66	2.47*E − *67	1.28*E − *66
	SCA	5.43*E + *03	3.79*E + *06	2.99*E + *05	6.84*E + *05	8.61*E + *08	8.53*E + *09	4.01*E + *09	1.68*E + *09
	SSA	0	1.01*E − *55	3.36*E − *57	1.84*E − *56	1.26*E − *248	1.51*E − *53	5.04*E − *55	2.76*E − *54
	MRFO	0	0	0	0	0	0	0	0
	LGMRFO	0	0	0	0	0	0	0	0

F5	BOA	2.30*E − *12	1.40*E − *11	7.28*E − *12	2.44*E − *12	1.28*E − *11	1.63*E − *11	1.43*E − *11	7.15*E − *13
	WOA	0	0	0	0	0	0	0	0
	SCA	3.95*E − *01	1.65*E + *00	1.12*E + *00	2.96*E − *01	1.57*E + *01	7.96*E + *01	5.01*E + *01	1.73*E + *01
	SSA	0	0	0	0	0	0	0	0
	MRFO	0	0	0	0	0	0	0	0
	LGMRFO	0	0	0	0	0	0	0	0

F6	BOA	0	1.34*E − *02	4.49*E − *05	2.45*E − *03	0	0	0	0
	WOA	0	0	0	0	0	0	0	0
	SCA	2.42*E + *02	4.29*E + *03	1.37*E + *03	1.02*E + *03	6.84*E + *04	3.47*E + *05	2.02*E + *05	8.54*E + *04
	SSA	0	0	0	0	0	0	0	0
	MRFO	0	0	0	0	0	0	0	0
	LGMRFO	0	0	0	0	0	0	0	0

F7	BOA	2.55*E − *15	1.75*E + *01	1.89*E + *00	4.82*E + *00	0	0	0	0
	WOA	0	7.77*E − *01	3.95*E − *02	1.58*E − *01	0	0	0	0
	SCA	6.39*E + *00	1.77*E + *01	1.41*E + *01	2.59*E + *00	5.87*E + *01	2.34*E + *02	1.80*E + *02	5.13*E + *01
	SSA	0	0	0	0	0	0	0	0
	MRFO	0	0	0	0	0	0	0	0
	LGMRFO	0	0	0	0	0	0	0	0

F8	BOA	0	3.59*E + *02	5.62*E + *01	1.28*E + *02	0	0	0	0
	WOA	0	0	0	0	0	0	0	0
	SCA	2.09*E + *02	2.27*E + *03	9.64*E + *02	5.04*E + *02	9.11*E + *04	3.56*E + *05	2.07*E + *05	6.99*E + *04
	SSA	0	0	0	0	0	0	0	0
	MRFO	0	0	0	0	0	0	0	0
	LGMRFO	0	0	0	0	0	0	0	0

F9	BOA	4.88*E + *01	4.90*E + *01	4.89*E + *01	3.31*E − *02	4.99*E + *02	4.99*E + *02	4.99*E + *02	2.75*E − *02
	WOA	4.76*E + *01	4.87*E + *01	4.82*E + *01	3.93*E − *01	4.96*E + *02	4.98*E + *02	4.97*E + *02	3.84*E − *01
	SCA	2.37*E + *06	2.57*E + *09	5.79*E + *08	5.52*E + *08	1.12*E + *11	3.54*E + *11	2.42*E + *11	5.69*E + *10
	SSA	4.13*E − *07	8.29*E − *03	1.60*E − *03	2.17*E − *03	1.62*E − *06	7.75*E − *03	1.35*E − *03	1.92*E − *03
	MRFO	4.27*E + *01	4.48*E + *01	4.37*E + *01	5.71*E − *01	4.94*E + *02	4.97*E + *02	4.96*E + *02	6.72*E − *01
	LGMRFO	4.29*E + *01	4.44*E + *01	4.35*E + *01	2.82*E − *01	4.91*E + *02	4.92*E + *02	4.91*E + *02	1.97*E − *01

F10	BOA	9.12*E − *12	1.41*E − *11	1.17*E − *11	1.21*E − *12	1.04*E − *11	1.47*E − *11	1.28*E − *11	1.21*E − *12
	WOA	3.03*E − *89	1.82*E − *69	6.35*E − *71	3.33*E − *70	5.05*E − *83	5.29*E − *69	2.95*E − *70	1.04*E − *69
	SCA	8.10*E + *00	2.94*E + *03	8.03*E + *02	8.46*E + *02	3.40*E + *04	1.82*E + *05	1.08*E + *15	3.80*E + *04
	SSA	0	1.71*E − *35	5.70*E − *37	3.11*E − *36	4.61*E − *241	1.18*E − *54	3.94*E − *56	2.16*E − *55
	MRFO	0	0	0	0	0	0	0	0
	LGMRFO	0	0	0	0	0	0	0	0

F11	BOA	2.11*E − *10	4.35*E − *09	1.49*E − *09	1.11*E − *09	7.82*E − *11	2.23*E − *09	4.66*E − *10	4.12*E − *10
	WOA	8.88*E − *16	7.99*E − *15	3.85*E − *15	2.65*E − *15	8.88*E − *16	1.51*E − *14	5.03*E − *15	3.37*E − *15
	SCA	2.04*E + *01	2.06*E + *01	2.05*E + *01	6.67*E − *01	2.08*E + *01	2.09*E + *01	2.09*E + *01	2.84*E − *02
	SSA	8.88*E − *16	8.88*E − *16	8.88*E − *16	0	8.88*E − *16	8.88*E − *16	8.88*E − *16	0
	MRFO	8.88*E − *16	8.88*E − *16	8.88*E − *16	0	8.88*E − *16	8.88*E − *16	8.88*E − *16	0
	LGMRFO	8.88*E − *16	8.88*E − *16	8.88*E − *16	0	8.88*E − *16	8.88*E − *16	8.88*E − *16	0

F12	BOA	1.37*E − *03	1.01*E − *01	2.97*E − *02	2.70*E − *02	5.91*E − *06	3.51*E − *04	7.83*E − *05	6.69*E − *05
	WOA	1.52*E − *47	5.89*E − *01	1.18*E − *01	1.90*E − *01	4.32*E − *57	4.26*E − *13	1.42*E − *14	7.78*E − *14
	SCA	1.27*E − *01	7.06*E − *01	3.55*E − *01	1.33*E − *01	3.43*E − *02	1.39*E − *01	7.27*E − *02	3.02*E − *02
	SSA	0	3.85*E − *16	2.02*E − *17	7.22*E − *17	0	3.62*E − *16	2.15*E − *17	7.20*E − *17
	MRFO	0	2.57*E − *13	3.21*E − *14	4.70*E − *14	0	3.76*E − *11	4.21*E − *12	1.01*E − *11
	LGMRFO	0	4.30*E − *13	9.43*E − *14	1.27*E − *13	0	0	0	0

**Table 4:** Comparison of some CEC2017 test suite Functions.

Function	Algorithm	Best	Worst	Average	Std. Deviation
CF2	BOA	61865.0516	94673.9128	83610.9	7252.6901
	WOA	181153.9155	432212.7775	276488.167	55312.8565
	SCA	47819.1154	168455.467	86410.2938	22263.7286
	SSA	62613.8174	88822.6913	76844.6378	5701.0961
	MRFO	9829.1363	31305.175	19475.5722	5541.5783
	**LGMRFO**	**3696.8277**	**25977.9711**	**12196.0016**	**5512.4282**

CF4	BOA	877.3537	967.557	910.4024	22.3843
	WOA	729.3879	1020.0647	864.4385	73.0595
	SCA	786.6671	876.3863	835.3316	26.4226
	SSA	670.135	847.6568	777.11	42.704
	MRFO	598.501	749.7332	657.6086	38.2902
	**LGMRFO**	**596.5108**	**742.7687**	**656.0086**	**32.1436**

CF7	BOA	1105.4266	1162.1825	1132.1944	15.1434
	WOA	1009.6932	1229.7966	1074.2146	51.6852
	SCA	1065.2217	1126.971	1096.4516	17.2106
	SSA	891.4775	1049.7886	992.9483	34.9974
	MRFO	873.6269	1002.9701	952.1615	34.1025
	**LGMRFO**	**881.5865**	**982.2495**	**934.2627**	**22.9263**

CF8	BOA	8895.1653	12920.2913	11075.1726	1016.128
	WOA	6526.484	24593.4414	11953.6288	4545.5098
	SCA	5801.305	12951.4022	9435.4069	2185.7205
	SSA	5377.5911	6872.3515	5815.5711	314.8259
	MRFO	2164.7351	7093.8441	4205.0785	1036.6014
	**LGMRFO**	**2152.914**	**5618.2209**	**3717.7776**	**748.5012**

CF10	BOA	6547.2791	13835.6547	9002.8469	2183.7801
	WOA	3775.3694	17919.2339	10044.4225	3734.4153
	SCA	2566.8743	5716.6906	3883.7186	870.4679
	SSA	1492.0962	4381.4378	2434.9342	820.455
	**MRFO**	**1165.9774**	**1315.8124**	**1240.9612**	**47.1172**
	LGMRFO	1164.0194	1259.8653	1201.5794	37.8005

CF15	BOA	4532.5588	12202.6872	7530.0974	1860.0716
	WOA	3091.6252	6343.4343	4183.5431	668.3028
	SCA	3391.0211	4496.9845	4182.2468	265.6575
	SSA	2430.5504	4058.9642	3139.6938	393.3999
	MRFO	2095.1895	3166.5832	2712.2462	317.7892
	**LGMRFO**	**2229.9637**	**3421.9934**	**2809.234**	**277.3386**

CF17	BOA	4956069.9615	195429416.0647	58482274.1537	48599692.6692
	WOA	466476.5171	41365723.3653	9301704.5173	10116889.255
	SCA	2977781.3915	38837593.3164	15400703.9766	9893645.6625
	SSA	81791.5292	12803104.8522	2438302.354	2728490.4502
	MRFO	41716.4756	962707.3555	254339.6966	203873.0355
	**LGMRFO**	**28304.0738**	**430158.1843**	**122081.5603**	**102567.4144**

CF20	BOA	2612.4543	2931.4312	2729.5077	205.2435
	WOA	2412.3452	2734.6753	2582.6538	66.6743
	SCA	2400.7732	2714.5564	2609.7752	76.453
	SSA	2423.4533	2612.1334	2543.1367	23.8764
	MRFO	2201.1145	2511.1134	2422.0052	16.0254
	**LGMRFO**	**2301.7768**	**2501.657**	**2404.667**	**13.1909**

CF24	BOA	4867.6438	7550.4929	6012.4665	605.8525
	WOA	3111.795	3356.4394	3222.9168	72.9402
	SCA	3305.9347	4349.4399	3601.44	268.54
	SSA	2937.7087	3081.5462	3001.3027	38.5158
	**MRFO**	**2885.7049**	**2942.7045**	**2900.6972**	**17.214**
	LGMRFO	2891.818	2979.9971	2932.3753	24.3826

**Table 5:** Wilcoxon rank sum test results for 50 and fixed dimensions.

F	MRFO	SSA	SCA	WOA	BOA
F1	NaN	1.21*E − *12	1.21*E − *12	1.21*E − *12	1.21*E − *12
F2	NaN	1.21*E − *12	1.21*E − *12	1.21*E − *12	1.21*E − *12
F3	NaN	1.66*E − *11	1.21*E − *12	1.21*E − *12	1.21*E − *12
F4	NaN	1.93*E − *10	1.21*E − *12	1.21*E − *12	1.21*E − *12
F5	NaN	NaN	1.21*E − *12	0.3337	1.21*E − *12
F6	NaN	NaN	1.21*E − *12	NaN	0.0013
F7	NaN	NaN	1.21*E − *12	NaN	1.21*E − *12
F8	NaN	NaN	1.21*E − *12	0.3337	1.95*E − *09
F9	0.0023	3.02*E − *11	3.02*E − *11	3.02*E − *11	3.02*E − *11
F10	NaN	1.66*E − *11	1.21*E − *12	1.21*E − *12	1.21*E − *12
F11	NaN	NaN	1.21*E − *12	2.17*E − *07	1.21*E − *12
F12	0.8877	0.2010	2.40*E − *11	2.42*E − *07	2.40*E − *11
F13	0.0419	3.46*E − *10	4.28*E − *11	3.86*E − *11	5.84*E − *11
F14	0.0080	4.09*E − *11	1.57*E − *11	1.57*E − *11	1.57*E − *11
F15	0.3128	3.02*E − *06	1.72*E − *12	1.72*E − *12	1.72*E − *12

**Table 6:** Wilcoxon rank sum test results for 500 dimensions.

F	MRFO	SSA	SCA	WOA	BOA
F1	NaN	5.77*E − *11	1.21*E − *12	1.21*E − *12	1.21*E − *12
F2	0.3337	5.77*E − *11	1.69*E − *14	1.69*E − *14	1.69*E − *14
F3	NaN	4.57*E − *12	1.21*E − *12	1.21*E − *12	1.21*E − *12
F4	NaN	4.57*E − *12	1.21*E − *12	1.21*E − *12	1.21*E − *12
F5	NaN	NaN	1.21*E − *12	NaN	1.21*E − *12
F6	NaN	NaN	1.21*E − *12	NaN	NaN
F7	NaN	NaN	1.21*E − *12	NaN	NaN
F8	NaN	NaN	1.21*E − *12	NaN	0.3337
F9	3.02*E − *11	3.02*E − *11	3.02*E − *11	3.02*E − *11	3.02*E − *11
F10	NaN	4.57*E − *12	1.21*E − *12	1.21*E − *12	1.21*E − *12
F11	NaN	NaN	1.21*E − *12	3.66*E − *08	1.21*E − *12
F12	1.27*E − *05	1.21*E − *12	1.21*E − *12	1.21*E − *12	1.21*E − *12

**Table 7:** Wilcoxon rank sum test results for 9 CEC2017 functions.

F	MRFO	SSA	SCA	WOA	BOA
CF2	1.5292*E − *05	3.0199*E − *11	3.0199*E − *11	3.0199*E − *11	3.0199*E − *11
CF4	0.9	4.1997*E − *10	3.0199*E − *11	4.0772*E − *11	3.0199*E − *11
CF7	0.040595	1.5581*E − *08	3.0199*E − *11	3.0199*E − *11	3.0199*E − *11
CF8	0.096263	5.4941*E − *11	3.0199*E − *11	3.0199*E − *11	3.0199*E − *11
CF10	0.00047138	3.0199*E − *11	3.0199*E − *11	3.0199*E − *11	3.0199*E − *11
CF15	0.26433	0.0015178	3.6897*E − *11	8.1527*E − *11	3.0199*E − *11
CF17	0.00065486	3.8249*E − *09	3.0199*E − *11	3.0199*E − *11	3.0199*E − *11
CF20	6.5991*E − *07	3.8249*E − *09	3.0199*E − *11	3.0199*E − *11	3.0199*E − *11
CF24	7.5991*E − *07	3.8249*E − *09	3.0199*E − *11	3.0199*E − *11	3.0199*E − *11

**Table 8:** Parameter setting for WSN coverage.

Parameters	Values
Region	50 m × 50 m
Number of nodes	30/35
Perceived radius	5 m
Communication radius	10 m

**Table 9:** Average coverage.

Algorithm	Average coverage/%			
	30 nodes	30 nodes initialization	35 nodes	35 nodes initialization
MRFO	82.79	63.36	89.24	67.47
LGMRFO	83.87	63.65	90.66	68.89

## Data Availability

The data used to support the study are available from the corresponding author upon request.
